# Qizhi Kebitong Formula Ameliorates Streptozocin-Induced Diabetic Osteoporosis through Regulating the PI3K/Akt/NF-*κ*B Pathway

**DOI:** 10.1155/2022/4469766

**Published:** 2022-08-21

**Authors:** Lulu Tian, Lu Ding, Guoqiang Wang, Yu Guo, Yunyun Zhao, Yuchi Wei, Xingquan Li, Wei Zhang, Jia Mi, Xiangyan Li, Zeyu Wang, Xiuge Wang

**Affiliations:** ^1^College of Chinese Medicine, Changchun University of Chinese Medicine, 130117, China; ^2^Jilin Ginseng Academy, Key Laboratory of Active Substances and Biological Mechanisms of Ginseng Efficacy, Ministry of Education, Jilin Provincial Key Laboratory of Bio-Macromolecules of Chinese Medicine, Changchun University of Chinese Medicine, Changchun, 130117 Jilin, China; ^3^Department of Endocrinology, The Affiliated Hospital to Changchun University of Chinese Medicine, Changchun 130021, China; ^4^Department of Scientific Research, Changchun University of Chinese Medicine, Changchun, China

## Abstract

**Background:**

Diabetic osteoporosis (DOP) is a progressive osteoblast dysfunction induced by high glucose, which has negative impacts on bone homeostasis. Qizhi Kebitong formula (QKF) is a traditional Chinese medicine (TCM) formula for treating DOP. However, its role in the protection of DOP has not been clarified yet. Here, we aimed to explore the potential mechanisms of QKF on DOP development via *in vivo* experiment.

**Methods:**

Network pharmacology was used to detect the key targets and signaling pathways of QKF on DOP. The effects of QKF on DOP were examined by the phenotypic characteristics, micro-CT, and hematoxylin-eosin (H&E) staining. The predicted targets and pathways were validated by a streptozocin- (STZ-) induced mouse model. Subsequently, the levels of the selected genes and proteins were analyzed using qRT-PCR and Western blot. Finally, AutoDock and PyMOL were used for molecular docking.

**Results:**

In this study, 90 active compounds and 2970 related disease targets have been found through network pharmacology. And QKF could improve the microstructures of femur bone mass, reduce inflammatory cell infiltration, and downregulate the levels of TNF-*α*, IKBKB, IL-6, and IL-1*β*. Moreover, the underlying effect of PI3K/Akt/NF-*κ*B pathways was also recommended in the treatment.

**Conclusion:**

Altogether, our findings suggested that QKF could markedly alleviate osteoblast dysfunction by modulating the key targets and PI3K/Akt/NF-*κ*B signaling pathway.

## 1. Introduction

Diabetic osteoporosis (DOP) is a common complication of diabetes, which primarily affects bone metabolism, joints, and kidney [1, 2]. DOP is a skeletal disorder characterized by a chronic high glucose, decreased bone mass, and damaged bone tissue [3–5]. With the increasing incidence of diabetes, DOP has become a systemic bone disease to increase bone brittleness, fracture risk, and impaired bone healing [6]. However, the pathogenesis of DOP has not been fully clarified. Notably, studies have shown that high glucose is a crucial determinant of DOP [7], especially increased diabetes-related pathological factors [8, 9]. Interestingly, inflammation is defined as one of the major pathological factors of DOP, which leads to bone loss [10], destroys the bone microenvironment, and inhibits bone formation [11, 12]. However, a series of DM-induced inflammation is often overlooked or underestimated, seriously affecting the quality of people's life in the later period [13]. Therefore, it is an urgent strategy to prevent the development of inflammation and find effective therapies for DOP.

Traditional Chinese medicine (TCM) has a long history in treating DOP and accumulated rich experience [14]. Qizhi Kebitong formula (QKF) is a classical TCM formula composed of seven TCMs, including Huang-qi (*Astragalus mongholicus* Bunge, Fabaceae, root), Ji-xue-teng (*Spatholobus suberectus* Dunn, Fabaceae, dry rattan stem), Huai-niu-xi (*Achyranthes bidentata* Blume, Amaranthaceae, root), Sang-zhi (*Morus alba* L., Moraceae, twig), Wei-ling-xian (*Clematis chinensis* Osbeck, Ranunculaceae, root), Xi-xian-cao (*Sigesbeckia orientalis* L., Asteraceae, aboveground part), and Quan-xie (scorpion, *Buthus martensi* Karsch, whole animal) in Table 1. Accumulating evidence demonstrates that QKF has beneficial effects on clinical observation, and the indispensable role of QKF has been widely accepted. But the mechanisms remain unknown.

In this study, the potential targets and protective pathways of QKF on DOP were screened *via* network pharmacology, and the results were verified in the mouse model. Then, we provided some insights with the possible molecular mechanisms of QKF on the clinical application for delaying DOP progression.

## 2. Materials and Methods

### 2.1. Preparation of QKF and Reagents

Herbal compounds of QKF were provided by a pharmacy of Jilin Provincial Hospital of Traditional Chinese Medicine (Changchun, China). All of the crude drugs (98 g, two-thirds are used clinically) were extracted in 1000 ml of distilled water three times (100°C, 1 h each time) to obtain the aqueous extract. The extracts were centrifuged at 3,500 rpm for 15 min, and the supernatant was freeze-dried to obtain the powdery extract of QKF, with a yield of 20% (13 g) for further experiments. According to dose translation of animal studies, the medium treatment concentration of a mouse is approximately equal to 3 g/kg/day; the low and high treatment concentrations are approximately equal to 1.5 g/kg/day and 6 g/kg/day, respectively. Streptozotocin (STZ) was purchased from Sigma-Aldrich (Shanghai, China). Antibodies against p-PI3K (AF3241, Affinity Biosciences, China), PI3K (ab227204, Abcam, USA), p-Akt (4058, Cell Signaling Technology, USA), Akt (ab179463, Abcam, USA), p-NF-*κ*B (3033, Cell Signaling Technology, USA), NF-*κ*B (ab16502, Abcam, USA), IL-6 (ab208113, Abcam, USA), IL-1*β* (ab254360, Abcam, USA), TNF-*α* (8184, Cell Signaling Technology, USA), IKBKB (15649-1AP, Proteintech, China), and GADPH (60004-1-1g, Proteintech, China) were used in this study.

### 2.2. Network Construction and Analysis

According to the pinyin form, “Huang-qi”, “Sang-zhi”, “Ji-xue-teng”, “Xi-xian-cao”, “Wei-ling-xian”, “Quan-xie”, and “Huai-niu-xi” were used as the keywords to search the active ingredients of XBC via the TCMSP (http://tcmspw.com/tcmsp.php) database. Meanwhile, DOP-associated targets were acquired from GeneCards (http://www.swisstargetprediction.ch/), OMIM, (https://OMIM.org/), PharmGKB, (https://www.pharmkb.org/), and DrugBank (https://www.drugbank.ca/). The protein-protein interaction (PPI) network was obtained from STRING (http://string-db.org/, v.11) with parameter conditions filtered by “Homo sapiens” (confidence score > 0.9) and visualized using Cytoscape 3.8.0. And Gene Ontology (GO) and Kyoto Encyclopedia of Genes and Genomes (KEGG) enrichment analyses were performed for the above targets.

### 2.3. Animals and Treatments

In this study, 48 male C57 BL/6 mice were used for animal experiments. They were purchased from Changchun Yisi Experimental Animal Co., Ltd. (license number SCXK (Beijing) 2016-0006) with the weight in 18~22 g. Meanwhile, all mice were approved for ethical use by the Experimental Animal Ethics Committee of Changchun University of Traditional Chinese Medicine (batch number 20190134). They were kept in the Animal Experimental Center of Changchun University of Traditional Chinese Medicine (Changchun, China). The ambient temperature is 18~22°C, and the humidity is 50~60%. Then, the mice were randomly divided into 5 groups (*n* = 8): control (Ctrl), STZ, QKF (1.5 g/kg), QKF (3 g/kg), and QKF (6 g/kg) groups. Except for the Ctrl group, all other mice were intraperitoneally injected with STZ 130 mg/kg. After 7 days, the tail of the mice was cut short to test the random blood glucose levels ≥ 300 mg/dl (16.7 mmol/l) which were considered to be diabetic.

### 2.4. Micro-Computed Tomography (Micro-CT) Scanning

The femurs were scanned with a high-resolution Quantum FX Micro-CT (PerkinElmer, Inc. Waltham, MA, USA), using the following settings: 80 *μ*A current, 90 kV voltage, 360° gantry rotation, 4 min scanning time, and 36 mm reconstructed visual field. The images were recombined via micro-CT, and the following parameters were recorded: bone mineral density (BMD), specific bone surface (BS/BV), trabecular separation (Tb.Sp), trabecular thickness (Tb.Th), bone volume over total volume (BV/TV), and connectivity density (Conn.D).

### 2.5. The Hematoxylin/Eosin (H&E) Staining

The exfoliated femurs were fixed using 4% formaldehyde, decalcified in EDTA glycerol solution, and embedded in paraffin. Paraffin sections were cut into the slices at 4 *μ*m thickness and stained with H&E. Images of the sections were captured using light microscopy (Olympus BX51, Japan) at 200x and 400x ratios, respectively.

### 2.6. Quantitative Real-Time PCR (qRT-PCR) Analysis

Total RNA was extracted from the femur tissues with a total RNA extraction kit (TIANGEN BIOTECH, China). Subsequently, the reverse transcription of 1 *μ*g total RNA into cDNA was conducted with the iScript cDNA synthesis kit (TIANGEN BIOTECH, China). The qRT-PCR assay was performed with a Bio-Rad CFX96 system, and the gene expressions of IKK, IL-1*β*, IL-6, and TNF-*α* were normalized to GAPDH. Relative mRNA levels were quantified using the 2^−ΔΔCt^ method. The mouse primer sequences are shown in Table 2.

### 2.7. Western Blotting Assay

Proteins were extracted from the femurs using RIPA lysis buffer (Beyotime, China) with phosphatase inhibitors and protease inhibitors. Protein quantification was measured using a BCA protein assay kit (Beyotime, China). The equivalent amount of protein was separated by 8%, 10%, or 12% SDS-PAGE and transferred to a PVDF membrane. The membrane was blocked with 5% BSA 1~2 h at room temperature. The antibodies against PI3K (1 : 1000), p-PI3K (1 : 1000), Akt (1 : 10000), p-Akt (1 : 1000), NF-*κ*B (1 : 2000), p-NF-*κ*B (1 : 1000), IKBKB (1 : 1000), TNF-*α* (1 : 1000), IL-1*β* (1 : 1000), IL-6 (1 : 1000), and GAPDH (1 : 5000) were added at 4°C overnight. After washing with 1× TBST, the membranes were further probed with the corresponding secondary antibody (1 : 5000) for 2 h at 18-25°C; the labeled protein bands were visualized using a BeyoECL Plus Kit (Beyotime, China). Image Lab software was used for semiquantitative analysis.

### 2.8. Molecular Docking

AutoDock software, version 4.2, was used for molecular docking. The composite targets were verified using the Lamarckian genetic algorithm; proteins and ligands were prepared using the AutoDock tool. The three-dimensional structure of the proteins was downloaded from the RCSB-PDB database (http://www.pdb.org), and the hydrogen atoms were added. We calculated the docking binding energy using the Auto tool. The docking diagrams of target proteins and molecules were performed by the PyMOL visualization software.

### 2.9. Statistical Analysis

All data were analyzed using GraphPad Prism 9.0. These data were compared with several groups by one-way ANOVA. For all statistical analysis, *p* < 0.05 was considered statistically significant.

## 3. Results

### 3.1. Screening of the Intersection Targets and Constructing a Series of Network

With OB ≥ 30% and DL ≥ 0.18 as screening parameters, 90 candidate compounds of QKF were found for further analysis (Table 3). Besides, 2970 potential targets of DOP were obtained from the four authoritative databases (Figure 1(a)). Through taking the intersection of 122 QKF targets and 2,970 DOP targets, 81 potential targets were obtained (Figure 1(b)). Subsequently, the intersection targets were inputted to Cytoscape software to build the network diagram with multicomponent and multitarget (Figure 1(c)). In addition, 81 potential targets were uploaded to the STRING database to construct the PPI network (Figure 1(d)). Among these nodes, PIK3CG, Akt1, and RELA were screened out with more relevance and biological functions in the PPI network (Figure 1(e)), suggesting that PIK3CG, Akt1, and RELA were the key genes, probably exhibiting therapeutic effect in DOP.

### 3.2. Functional Enrichment Analysis

To investigate the potential mechanisms, the 1660 biological processes (BP), 24 cellular components (CC), and 104 molecular functions (MF) were performed using the DAVID database. Moreover, the top 15 results were selected with the *p* value from small to large (Figure 2(a) and Table 4). KEGG enrichment analysis obtained 128 results. Subsequently, we selected the top 50 according to the *p* value for further analysis (Figure 2(b)). Notably, previous studies indicated the osteogenic differentiation through activating the PI3K/Akt pathway, connected with the multitarget and multicomponent. Among these enriched pathways, PI3K/Akt played an important role in DOP; the predictive targets are shown in Figure 2(c).

### 3.3. Effect of QKF on the General Features of STZ-Induced Mice

In order to determine the effect of QKF on DOP, we established a STZ-induced mouse model and compared disease evolution in groups (Figure 3). After administration of QKF for 4 months, blood glucose levels of STZ-induced mice were significantly higher (Figure 3(a)), while body weight was significantly lower (Figure 3(b)). The results demonstrated that the blood glucose of mice increased sharply, which consumed a lot of fat in the body. And compared to the Ctrl group, the weight of mice in STZ and QKF groups was decreased significantly. Meanwhile, the trabecular bone at distal femoral metaphysis was assessed by HE staining (Figure 3(c)); obvious bone loss was observed in STZ-induced mice compared with the Ctrl group, which was gradually mitigated with the increasing dose of QKF. The femurs of normal mice scattered pink trabecular bones, and the number of trabecular bones was reduced in STZ-induced mice. Furthermore, the profiles of 3D images (Figure 3(d)) clearly exhibited the breakage of cancellous bone of diabetic mice, and the 3D bone biological parameters (Figures 3(e)–3(j)) quantitatively reflected the significant reduction in Conn.D (*p* < 0.001), BMD (*p* < 0.001), BV/TV (*p* < 0.01), BS/TV (*p* < 0.001), and Tb.Th (*p* < 0.01) in the STZ group, while Tb.Sp was significantly increased. However, after the treatment of QKF for 4 months, improved bone mass of trabecular bone and reversed changes of biological parameters indicated the potential therapeutic efficacy of QKF on DOP.

### 3.4. QKF Improves STZ-Induced Mouse Inflammation

DOP is an inflammatory response caused by high blood glucose [15]. To validate that QKF could reduce the inflammatory expression of STZ-induced mice, we used qRT-PCR and Western blot to determine changes in mRNA and protein levels (Figure 4). The qRT-PCR results indicated that the mRNA levels of TNF-*α*, IKK, IL-6, and IL-1*β* were significantly downregulated after administration (Figure 4(a)). Meanwhile, Western blot results demonstrated that QKF had a similar inhibitory effect at the protein levels (Figures 4(b) and 4(c)). Above all, these results indicate that QKF could attenuate inflammation in STZ-induced mice.

### 3.5. QKF Mediated Inflammation through the PI3K/Akt/NF-*κ*B Pathway

Based on the network pharmacological analysis, the PI3K/Akt signaling pathway may be predicted as a potential mechanism of QKF for DOP protection. Meanwhile, NF-*κ*B was a key downstream factor of the PI3K/Akt pathway, which was closely related to the regulation of glucose and lipid metabolism [16]. Therefore, we explored the PI3K/Akt/NF-*κ*B signaling pathway as the potential mechanism of QKF for experimental verification. After administration of QKF, the protein levels of p-PI3K/PI3K and p-Akt/Akt were further upregulated compared with the STZ group, while p-NF-*κ*B/NF-*κ*B was downregulated (Figure 5). The results indicated that PI3K/Akt/NF-*κ*B signaling could regulate the protective effects of QKF on DOP.

### 3.6. Molecular Docking Analysis

To further explore the effect of the 3 major compounds of QKF on the 7 potential targets, including PI3K, Akt1, RELA, IKBKB, IL-1*β*, TNF-a, and IL-6, the binding energies were determined by molecular docking (Figure 6). Firstly, kaempferol and baicalein had a strong binding ability with PI3K, so they would be a potential bioactive compound of QKF on DOP (Figure 6(a)). Akt1 had a stronger binding energy with all compounds (Figure 6(b)). The strongest binding energy was as high as -10.2 kcal/mol. Interestingly, quercetin, kaempferol, and baicalein had the same binding power with RELA and IL-6 (Figures 6(c) and 6(g)). It means that RELA and IL-6 have the best binding force with the above components. Meanwhile, IKBKB and baicalein, IL-1*β* and quercetin, and TNF-*α* and quercetin have a stronger binding force (Figures 6(d)–6(f)). Above, quercetin, kaempferol, and baicalein played an important role in QKF. Although they have higher binding force with inflammatory factors, the pharmacological effects of these active compounds in regulating key targets needed to be further verified.

## 4. Discussion

In this study, we performed network pharmacology, animal experiments, and molecular docking to explore the active compositions and molecular mechanisms of QKF in the treatment of DOP. The potential targets and enrichment pathways were predicted by network pharmacology. Histopathological staining and micro-CT imaging confirmed the therapeutic effect of QKF on the STZ-induced mouse model. qRT-PCR and Western Blot confirmed that QKF could mediate inflammation through the PI3K/Akt/NF-*κ*B pathway. In summary, this study demonstrated for the first time that QKF mediated inflammation through the PI3K/Akt/NF-*κ*B pathway, thereby improving bone mass of trabecular bone and reversing the changes of biological parameters in the STZ-induced mouse model.

Based on the TCM theory, seven drugs of QKF were formed for clinical application of DOP-related diseases [17]. Among these drugs, HQ (qi-tonifying), JXT (blood-activating), HNX (kidney-invigorating), and WLX, SZ, and XXC (dredging collateral) were used for the treatment of DOP [18–20]. A large number of reports have focused on bones and kidneys [21]; kidney weakness and blood stasis were the main causes of DOP [22]. Therefore, the kidney-nourishing herbs used for the treatment of DOP have aroused concerns [23]. HNX and WLX could tonify the kidney [24], which was deemed as one of the effective methods to alleviate DOP [25]. Furthermore, SZ and XXC had the ability to tonify the kidney and strengthen muscle and bone [26]. Above all, TCM has a series of effects on DOP [27], and it could improve the clinical symptoms of patients, which was worthy of clinical promotion [28]. At the same time, a previous study suggested that quercetin not only promoted the differentiation activity of osteoblasts but also inhibited the absorption activity of osteoclasts, thereby increasing the expression of osteogenic markers [29]. Kaempferol has a significant anti-inflammatory benefits, including promoting osteoblast proliferation, differentiation, and bone formation [30]. Previous studies suggested that baicalin could promote osteogenic differentiation by regulating protein kinases and transcription factors [31]. In sum, the compounds of QKF could provide an alternative strategy to prevent bone loss.

According to reports, trabecular bone loss was one of the common pathological processes occurring in DOP mice. To evaluate the effects of QKF for the treatment of DOP, we assessed trabecular architectural parameters using 3D micro-CT images. The results suggested that QKF could prevent the loss of bone mass induced by DOP and restore the trabecular connectivity by increasing BMD and Conn.D. Moreover, compared with the STZ group, the parameters of Tb.Th, BS/BV, and BV/TV in the QKF group increased significantly, while that of Tb.Sp was inhibited. Treatment of STZ-induced mice with QKF markedly increased trabecular BMD and improved trabecular bone and enhanced trabecular bone area.

In the present study, QKF treatment significantly decreased the mRNA and protein levels of a series of inflammatory factors, including IL-6, TNF-*α*, IKBKB, and IL-1*β* in the STZ-induced mouse model, which contributed to the improvement of DOP. However, QKF mediated inflammation through the PI3K/Akt/NF-*κ*B pathway; the relevant key targets were also proven to induce antioxidation, anti-inflammation, and immune regulation. Among them, Akt was identified as a unique signaling intermediate in bone homeostasis that controlled the differentiation of osteoblasts and osteoclasts, which was a direct downstream target of PI3K to inhibit the release of inflammatory factors [32–36]. Moreover, NF-*κ*B was also a key downstream factor of the PI3K/Akt pathway, which enhanced the degree of inflammatory response and promoted the differentiation of osteoclast precursors [37, 38]. Meanwhile, the PI3K/Akt signaling pathway not only affects inflammatory factors such as NF-*κ*B and TNF-*α* but also induced the inflammatory reaction in the internal environment of the body. Furthermore, the differentiation of osteoblasts was regulated by TNF-*α*, which was the earliest inflammatory mediator produced in response to oxidative stress and promoted the production of inflammatory cytokines to promote osteoblast apoptosis [39, 40]. In addition, accumulating studies have revealed that the expressions of core targets, including Akt1, TNF-*α*, IL-6, and RELA, made the vital functions in regulating inflammatory response [41, 42]. We have verified that QKF could regulate the key targets and PI3K/Akt/NF-*κ*B signaling pathway to explain the molecular mechanism of QKF treatment on DOP.

## 5. Conclusion

In summary, QKF could recuperate the bone loss and improve bone mass of trabecular bone in STZ-induced mouse models by downregulating the expression of IL-6, TNF-*α*, IKBKB, and IL-1*β* to alleviate the inflammation. The results might be mediated by the PI3K/Akt/NF-*κ*B pathway based on the prediction from network pharmacology and experiment validation. This study may provide new insights into the molecular mechanisms of QKF in the treatment of DOP.

## Figures and Tables

**Figure 1:** Construction and analysis of the network pharmacology. (a) Disease-related targets. (b) The interactive targets of QKF and DOP. (c) The drug-compound-target-disease network. (d) PPI network and cluster analysis of the potential targets. (e) PPI network of significant genes was extracted.

**Figure 2:** (a) GO enrichment analysis. The top 15 BP terms, CC terms, and MF terms are shown as a bubble chart according to the -log *p* value. The colors represent the different adjusted *p* value < 0.05, and the abscissa represents the number of target genes. The smaller *p* value represents higher significance. (b) The top 50 entries of KEGG pathway analysis are ordered according to the -lg *p* value. The redder color represents more obvious enrichment. (c) The PI3K/Akt signaling pathway modified from hsa04151. Red represents the targets of QKF.

**Figure 3:** Effect of QKF on the general features of STZ-induced mice. (a) Blood glucose. (b) Body weight. (c) Representative HE staining images of the trabecular bone. (d) Three-dimensional (3D) micro-CT images of femur. Trabecular bone biological parameters: (e) BMD, (f) BS/TV, (g) BV/TV, (h) Conn.D, (i) Tb.Sp, and (j) Tb.Th. The results are triplicates from a representative experiment. ^∗^*p* < 0.05, ^∗∗^*p* < 0.01, and ^∗∗∗^*p* < 0.001 vs. STZ group. ^##^*p* < 0.01 and ^###^*p* < 0.001 vs. Ctrl group.

**Figure 4:** QKF improves STZ-induced mouse inflammation. (a) qRT-PCR method was used to detect the mRNA levels of TNF-*α*, IKK, IL-6, and IL-1*β*. (b, c) Western blot method was used to detect the protein levels of TNF-*α*, IKBKB, IL-6, and IL-1*β*. Data were expressed as mean ± SD (*n* = 8). ^∗^*p* < 0.05, ^∗∗^*p* < 0.01, and ^∗∗∗^*p* < 0.001 vs. STZ group. ^#^*p* < 0.05, ^##^*p* < 0.01, and ^###^*p* < 0.001 vs. Ctrl group.

**Figure 5:** QKF mediated inflammation through the PI3K/Akt/NF-*κ*B pathway. Western blot method was used to detect the protein levels of (b) p-PI3K/PI3K, (c) p-Akt/Akt, and (d) p-NF-*κ*B/NF-*κ*B. ^∗^*p* < 0.05 and ^∗∗∗^*p* < 0.001 vs. STZ group. ^#^*p* < 0.05 and ^###^*p* < 0.001 vs. Ctrl group.

**Figure 6:** The protein-ligand of the docking simulation. Simulated molecular docking of (a) PI3K with quercetin, kaempferol, and baicalein. (b) Akt1 with quercetin, kaempferol, and baicalein. (c) RELA with quercetin, kaempferol, and baicalein. (d) IKBKB with quercetin, kaempferol, and baicalein. (e) IL-1*β* with quercetin, kaempferol, and baicalein. (f) TNF-*α* with quercetin, kaempferol, and baicalein. (g) IL-6 with quercetin, kaempferol, and baicalein.

**Table 1:** The compositions of QKF.

Chinese pinyin name	Taxonomy name	Abbr.	Family	Weight (g)	Part used
Huang-qi	*Astragalus mongholicus* Bunge	HQ	Fabaceae	30	Root
Ji-xue-teng	*Spatholobus suberectus* Dunn	JXT	Fabaceae	15	Dry rattan stem
Huai-niu-xi	*Achyranthes bidentata* Blume	HNX	Amaranthaceae	10	Root
Sang-zhi	*Morus alba* L.	SZ	Moraceae	20	Twig
Wei-ling-xian	*Clematis chinensis* Osbeck	WLX	Ranunculaceae	15	Root
Xi-xian-cao	*Sigesbeckia orientalis* L.	XXC	Asteraceae	20	Aboveground part
Quan-xie	Scorpion	QX	*Buthus martensi* Karsch	5	Dry body

**Table 2:** Primer sequences of qRT-PCR in mouse.

Target	Forward (5′ to 3′)	Reverse (5′ to 3′)
IKK	GGCAGAAGAGCGAAGTGGACATC	CCAGCCGTTCAGCCAAGACAC
IL-1*β*	GAAATGCCACCTTTTGACAGTG	TGGATGCTCTCATCAGGACAG
IL-6	CCAAGAGGTGAGTGCTTCCC	CTGTTGTTCAGACTCTCTCCCT
TNF-*α*	TGAGCACAGAAAGCATGATCC	GCCATTTGGGAACTTCTCATC
GAPDH	AGGTCGGTGTGAACGGATTTG	TGTAGACCATGTAGTTGAGGTCA

**Table 3:** The 90 active components of QKF were screened from the TCMSP database.

Drug	MOL_ID	Molecule name	OB (%)	DL
*Astragalus mongholicus* Bunge (Huang-qi)	MOL000211	Mairin	55.38	0.78
	MOL000239	Jaranol	50.83	0.29
	MOL000295	Alexandrin	20.63	0.63
	MOL000296	Hederagenin	36.91	0.75
	MOL000033	(3S,8S,9S,10R,13R,14S,17R)-10,13-Dimethyl-17-[(2R,5S)-5-propan-2-yloctan-2-yl]-2,3,4,7,8,9,11,12,14,15,16,17-dodecahydro-1H-cyclopenta[a]phenanthren-3-ol	36.23	0.78
	MOL000354	Isorhamnetin	49.6	0.31
	MOL000371	3,9-Di-O-methylnissolin	53.74	0.48
	MOL000374	5′-Hydroxyiso-muronulatol-2′,5′-di-O-glucoside	41.72	0.69
	MOL000378	7-O-Methylisomucronulatol	74.69	0.3
	MOL000379	9,10-Dimethoxypterocarpan-3-O-*β*-D-glucoside	36.74	0.92
	MOL000380	(6aR,11aR)-9,10-Dimethoxy-6a,11a-dihydro-6H-benzofurano[3,2-]chromen-3-ol	64.26	0.42
	MOL000387	Bifendate	31.1	0.67
	MOL000392	Formononetin	69.67	0.21
	MOL000398	Isoflavanone	109.99	0.3
	MOL000417	Calycosin	47.75	0.24
	MOL000422	Kaempferol	41.88	0.24
	MOL000433	FA	68.96	0.71
	MOL000438	(3R)-3-(2-Hydroxy-3,4-dimethoxyphenyl)chroman-7-ol	67.67	0.26
	MOL000439	Isomucronulatol-7,2′-di-O-glucosiole	49.28	0.62
	MOL000440	Isomucronulatol-7,2′-di-O-glucosiole_qt	23.42	0.79
	MOL000442	1,7-Dihydroxy-3,9-dimethoxy pterocarpene	39.05	0.48
	MOL000098	Quercetin	46.43	0.28
*Morus alba* L. (Sang-zhi)	MOL000422	Kaempferol	41.88	0.24
	MOL000729	Oxysanguinarine	46.97	0.87
	MOL000737	Morin	46.23	0.27
*Spatholobus suberectus* Dunn (Ji-xue-teng)	MOL000392	Formononetin	69.67	0.21
	MOL000471	Aloe-emodin	83.38	0.24
	MOL000492	(+)-Catechin	54.83	0.24
	MOL000417	Calycosin	47.75	0.24
	MOL000006	Luteolin	36.16	0.25
	MOL000461	3,7-Dihydroxy-6-methoxy-dihydroflavonol	43.8	0.26
	MOL000483	(Z)-3-(4-Hydroxy-3-methoxy-phenyl)-N-[2-(4-hydroxyphenyl)ethyl]acrylamide	118.35	0.26
	MOL000468	8-o-Methylreyusi	70.32	0.27
	MOL000501	Consume close grain	68.12	0.27
	MOL000502	Cajinin	68.8	0.27
	MOL000497	Licochalcone A	40.79	0.29
	MOL000490	Petunidin	30.05	0.31
	MOL000507	Psi-baptigenin	70.12	0.31
	MOL000503	Medicagol	57.49	0.6
	MOL000491	Augelicin	37.5	0.66
	MOL000470	8-C-*α*-L-Arabinosylluteolin	35.54	0.66
	MOL000493	Campesterol	37.58	0.71
	MOL000296	Hederagenin	36.91	0.75
	MOL000358	Beta-sitosterol	36.91	0.75
	MOL000449	Stigmasterol	43.83	0.76
	MOL000033	(3S,8S,9S,10R,13R,14S,17R)-10,13-Dimethyl-17-[(2R,5S)-5-propan-2-yloctan-2-yl]-2,3,4,7,8,9,11,12,14,15,16,17-dodecahydro-1H-cyclopenta[a]phenanthren-3-ol	36.23	0.78
	MOL000469	3-Hydroxystigmast-5-en-7-one	40.93	0.78
*Sigesbeckia orientalis* L. (Xi-xian-cao)	MOL004180	Coronaridine	34.97	0.68
	MOL000296	Hederagenin	36.91	0.75
	MOL000358	Beta-sitosterol	36.91	0.75
	MOL004179	Vernolic acid	37.63	0.19
	MOL000449	Stigmasterol	43.83	0.76
	MOL004172	(1R)-1-[(2S,4aR,4bS,7R,8aS)-7-Hydroxy-2,4b,8,8-tetramethyl-4,4a,5,6,7,8a,9,10-octahydro-3H-phenanthren-2-yl]ethane-1,2-diol	46.7	0.31
	MOL004184	Siegesesteric acid II	51.98	0.48
	MOL004177	15alpha-Hydroxy-ent-kaur-16-en-19-oic acid	58.73	0.38
	MOL004185	Siegesmethyletheric acid	60.72	0.43
*Clematis chinensis* Osbeck (Wei-ling-xian)	MOL001663	(4aS,6aR,6aS,6bR,8aR,10R,12aR,14bS)-10-Hydroxy-2,2,6a,6b,9,9,12a-heptamethyl-1,3,4,5,6,6a,7,8,8a,10,11,12,13,14b-tetradecahydropicene-4a-carboxylic acid	32.03	0.76
	MOL002372	(6Z,10E,14E,18E)-2,6,10,15,19,23-Hexamethyltetracosa-2,6,10,14,18,22-hexaene	33.55	0.42
	MOL005598	Embinin	33.91	0.73
	MOL000358	Beta-sitosterol	36.91	0.75
	MOL005594	ClematosideA′_qt	37.51	0.76
	MOL005603	Heptyl phthalate	42.26	0.31
	MOL000449	Stigmasterol	43.83	0.76
*Achyranthes bidentata* Blume (Huai-niu-xi)	MOL001006	Poriferasta-7,22E-dien-3beta-ol	42.98	0.76
	MOL012461	28-Norolean-17-en-3-ol	35.93	0.78
	MOL012505	Bidentatoside,ii_qt	31.76	0.59
	MOL012537	Spinoside A	41.75	0.4
	MOL012542	*β*-Ecdysterone	44.23	0.82
	MOL001454	Berberine	36.86	0.78
	MOL001458	Coptisine	30.67	0.86
	MOL000173	Wogonin	30.68	0.23
	MOL002643	Delta 7-stigmastenol	37.42	0.75
	MOL002714	Baicalein	33.52	0.21
	MOL002776	Baicalin	40.12	0.75
	MOL002897	Epiberberine	43.09	0.78
	MOL000358	Beta-sitosterol	36.91	0.75
	MOL003847	Inophyllum E	38.81	0.85
	MOL000422	Kaempferol	41.88	0.24
	MOL004355	Spinasterol	42.98	0.76
	MOL000449	Stigmasterol	43.83	0.76
	MOL000785	Palmatine	64.6	0.65
	MOL000085	Beta-daucosterol_qt	36.91	0.75
	MOL000098	Quercetin	46.43	0.28
*Scorpion* (Quan-xie)	MOL011455	20-Hexadecanoylingenol	32.7	0.65
	MOL000953	Cholesterol	37.87	0.68
	MOL002223	Taurine	24.37	0.21
	MOL002156	Trimethylamine	59.98	0.18
	MOL000860	Stearic acid	17.83	0.14
	MOL002223	Taurine	24.37	0.01
	MOL000069	Palmitic acid	19.3	0.1

**Table 4:** GO enrichment analysis of QKF.

Ontology	ID	Description	*p* value	*p*.adjust	GeneID	Count
Biological process (BP)	GO:0048545	Response to steroid hormone	2.00*E* − 21	6.65*E* − 18	PGR/AR/ESR2/NCOA2/NR3C2/NCOA1/ESR1/RELA/RXRB/BCL2/CASP3/ICAM1/GSTP1/EGFR/CCND1/FOS/CASP9/IL6/TP63/CAV1/PARP1/MDM2/FOSL1	23
	GO:0062197	Cellular response to chemical stress	4.92*E* − 21	8.18*E* − 18	PPARG/AKR1B1/RELA/BCL2/CASP3/MAPK8/CYP1B1/ALOX5/GSTP1/SLC2A4/EGFR/FOS/IL6/HIF1A/CAV1/NOS3/HSPB1/NFE2L2/NQO1/PARP1/MDM2/CYCS/CD36	23
	GO:1901654	Response to ketone	3.35*E* − 19	3.71*E* − 16	AR/NCOA2/NCOA1/PPARG/AKR1B1/F7/RELA/ICAM1/AHR/EGFR/CCND1/FOS/CASP9/ELK1/CAV1/PARP1/PRKCE/FOSL1	18
	GO:0006979	Response to oxidative stress	1.09*E* − 18	9.05*E* − 16	PTGS1/RELA/BCL2/CASP3/MAPK8/CYP1B1/ALOX5/GSTP1/EGFR/FOS/IL6/HIF1A/NOS3/HSPB1/NFE2L2/NQO1/PARP1/MDM2/APP/FOSL1/CYCS/SP1/CD36	23
	GO:0042493	Response to drug	1.55*E* − 17	1.03*E* − 14	NCOA1/PPARG/F7/RELA/ADRA1A/BCL2/CASP3/CYP3A4/CYP1A1/ICAM1/EGFR/CCND1/FOS/POR/MYC/CCNB1/NFE2L2/CHEK2/MDM2/FOSL1/DRD2	21
	GO:0034599	Cellular response to oxidative stress	8.36*E* − 16	4.44*E* − 13	RELA/BCL2/MAPK8/CYP1B1/ALOX5/GSTP1/EGFR/FOS/IL6/HIF1A/NOS3/HSPB1/NFE2L2/NQO1/PARP1/MDM2/CYCS/CD36	18
	GO:0010038	Response to metal ion	9.35*E* − 16	4.44*E* − 13	BCL2/CASP3/MAPK8/CYP1A1/ICAM1/EGFR/CCND1/FOS/CASP9/CASP8/HIF1A/CAV1/CCNB1/NFE2L2/NQO1/PARP1/MDM2/APP/DRD2	19
	GO:0009636	Response to toxic substance	8.72*E* − 15	3.62*E* − 12	PTGS1/BCL2/CYP1A1/CYP1B1/GSTP1/AHR/GSTM1/FOS/NOS3/CCNB1/NFE2L2/NQO1/PON1/MDM2/CD36/DRD2	16
	GO:0009314	Response to radiation	3.52*E* − 14	1.30*E* − 11	RELA/BCL2/CASP3/MAPK8/ICAM1/EGFR/CCND1/FOS/CASP9/ELK1/HIF1A/MYC/PARP1/COL3A1/CHEK2/MDM2/APP/TYR/DRD2	19
	GO:0000302	Response to reactive oxygen species	6.77*E* − 14	2.25*E* − 11	RELA/BCL2/CASP3/MAPK8/CYP1B1/GSTP1/EGFR/FOS/IL6/NOS3/NFE2L2/NQO1/MDM2/FOSL1/CD36	15
Cell component (CC)	GO:0045121	Membrane raft	1.05*E* − 08	1.31*E* − 06	ADRA1A/CASP3/ICAM1/SELE/SLC2A4/EGFR/CASP8/CAV1/NOS3/CTSD/APP/CD36	12
	GO:0098857	Membrane microdomain	1.09*E* − 08	1.31*E* − 06	ADRA1A/CASP3/ICAM1/SELE/SLC2A4/EGFR/CASP8/CAV1/NOS3/CTSD/APP/CD36	12
	GO:0098589	Membrane region	1.67*E* − 08	1.34*E* − 06	ADRA1A/CASP3/ICAM1/SELE/SLC2A4/EGFR/CASP8/CAV1/NOS3/CTSD/APP/CD36	12
	GO:0005667	Transcription regulator complex	1.05*E* − 06	6.29*E* − 05	PPARG/RELA/RXRB/AHR/CCND1/FOS/RB1/HIF1A/PARP1/RUNX2/SP1	11
	GO:0005901	Caveola	0.000373551	0.016511501	ADRA1A/SELE/CAV1/NOS3	4
	GO:0031983	Vesicle lumen	0.000420556	0.016511501	ALOX5/GSTP1/EGFR/VEGFA/CTSD/IGF2/APP	7
	GO:0090575	RNA polymerase II transcription regulator complex	0.000549681	0.016511501	PPARG/RXRB/FOS/RB1/HIF1A	5
	GO:0031091	Platelet alpha granule	0.000554949	0.016511501	VEGFA/IGF2/APP/CD36	4
	GO:0005641	Nuclear envelope lumen	0.000746032	0.016511501	ALOX5/APP	2
	GO:0000307	Cyclin-dependent protein kinase holoenzyme complex	0.000749375	0.016511501	CCND1/RB1/CCNB1	3
Molecular functions (mf)	GO:0140297	DNA-binding transcription factor binding	1.46*E* − 13	5.42*E* − 11	NCOA2/NCOA1/ESR1/PPARG/GSK3B/RELA/BCL2/FOS/RB1/NFKBIA/HIF1A/MYC/HSPB1/NFE2L2/PARP1/RUNX2/SP1	17
	GO:0004879	Nuclear receptor activity	1.27*E* − 12	1.57*E* − 10	PGR/AR/ESR2/NR3C2/ESR1/PPARG/RXRB/AHR/NR1I3	9
	GO:0098531	Ligand-activated transcription factor activity	1.27*E* − 12	1.57*E* − 10	PGR/AR/ESR2/NR3C2/ESR1/PPARG/RXRB/AHR/NR1I3	9
	GO:0061629	RNA polymerase II-specific DNA-binding transcription factor binding	1.04*E* − 11	9.58*E* − 10	NCOA2/NCOA1/ESR1/PPARG/GSK3B/RELA/FOS/RB1/NFKBIA/HIF1A/HSPB1/NFE2L2/PARP1/SP1	14
	GO:0003707	Steroid hormone receptor activity	9.04*E* − 08	5.81*E* − 06	PGR/ESR2/NR3C2/ESR1/RXRB	5
	GO:0001221	Transcription cofactor binding	9.41*E* − 08	5.81*E* − 06	PGR/AR/ESR1/RELA/AHR/NFE2L2	6
	GO:0044389	Ubiquitin-like protein ligase binding	1.38*E* − 07	7.27*E* − 06	GSK3B/RELA/BCL2/EGFR/RB1/NFKBIA/CASP8/HIF1A/CCNB1/CHEK2/MDM2	11
	GO:0001223	Transcription coactivator binding	1.62*E* − 07	7.47*E* − 06	PGR/AR/ESR1/RELA/AHR	5
	GO:0005496	Steroid binding	4.30*E* − 07	1.71*E* − 05	PGR/AR/ESR2/NR3C2/ESR1/CYP3A4/CAV1	7
	GO:0097153	Cysteine-type endopeptidase activity involved in apoptotic process	4.63*E* − 07	1.71*E* − 05	CASP3/CASP9/CASP8/CASP7	4

## Data Availability

The datasets used and/or analyzed during the current study are available from the corresponding author on reasonable request.

## Additional Points

*Strengths and Limitations*. These results demonstrate that QKF inhibits high glucose-induced osteoporosis by regulating the key targets and PI3K/Akt/NF-*κ*B signaling pathway. The potential mechanisms of QKF on DOP development need to be further confirmed by multiple targets and multiple pathways.
